# Automatic Diagnosis of Alzheimer's Disease and Mild Cognitive Impairment Based on CNN + SVM Networks with End-to-End Training

**DOI:** 10.1155/2021/9121770

**Published:** 2021-08-13

**Authors:** Zhe Huang, Minglang Sun, Chengan Guo

**Affiliations:** School of Information and Communication Engineering, Dalian University of Technology, Dalian 116023, China

## Abstract

Alzheimer's disease (AD) is an irreversible neurodegenerative disease, and, at present, once it has been diagnosed, there is no effective curative treatment. Accurate and early diagnosis of Alzheimer's disease is crucial for improving the condition of patients since effective preventive measures can be taken in advance to delay the onset time of the disease. ^18^F-Fluorodeoxyglucose positron emission tomography (^18^F-FDG PET : PET) is an effective biomarker of the symptom of AD and has been used as medical imaging data for diagnosing AD. Mild cognitive impairment (MCI) is regarded as an early symptom of AD, and it has been shown that MCI also has a certain biomedical correlation with PET. In this paper, we explore how to use 3D PET images to realize the effective recognition of MCI and thus achieve the early prediction of AD. This problem is then taken as the classification of three categories of PET images, including MCI, AD, and NC (normal controls). In order to get better classification performance, a novel network model is proposed in the paper based on 3D convolution neural networks (CNN) and support vector machines (SVM) by utilizing both the excellent abilities of CNN in feature extraction and SVM in classification. In order to make full use of the optimal property of SVM in solving binary classification problems, the three-category classification problem is divided into three binary classifications, and each binary classification is being realized with a CNN + SVM network. Then, the outputs of the three CNN + SVM networks are fused into a final three-category classification result. An end-to-end learning algorithm is developed to train the CNN + SVM networks, and a decision fusion algorithm is exploited to realize the fusion of the outputs of three CNN + SVM networks. Experimental results obtained in the work with comparative analyses confirm the effectiveness of the proposed method.

## 1. Introduction

Alzheimer's disease (AD), as a chronic neurodegenerative disease characterized by irreversible loss of neurons and genetically complex disorder, is often found in the elderly people [1]. Unfortunately, there is no effective curative treatment to reverse AD at present due to the irreversible brain atrophy. Thus, the early diagnosis of AD and its prodromal stage, i.e., mild cognitive impairment (MCI), is vital for patient care and slowing down progressive deterioration [2]. However, patients with MCI only have subtle typical changes, so the accurate diagnosis of MCI is still a difficult problem in early AD diagnosis.

Since the metabolic rate and structure of the brain change accordingly with the progression of AD, the positron emission tomography (PET) is usually utilized to quantify the changes and further applied for computer-aided diagnosis (CAD) of AD [3–5]. In computer-aided AD diagnosis, various pattern recognition-based methods have been employed to predict AD and MCI, and these methods can be roughly divided into two steps, feature extraction and classification. The feature extraction step is to extract discriminative features from the PET images, and the classification step is to get prediction results according to the extracted features. Gray et al. [6] used two support vector machine (SVM) classifiers to identify NC vs. MCI and NC vs. AD, in which the SVMs are trained with the features of mean signal intensity in the region of native MRI-space of each subject. Garali et al. [7] proposed a novel brain region validity ranking method to separate AD from healthy controls, where SVM and random forest are employed for classification with the features obtained from selected 21 regions. Silveira and Marques [8] developed a boosting classification method that mixed a group of simple classifiers to perform feature selection and segmentation. Cabral and Silveira [9] used different ensemble classifiers based on SVM and random forest to extract diverse features on different sets of brain voxels for classification. Lu et al. [10] extracted three groups of spatial features from PET images and proposed a semisupervised classification method based on random manifold learning with affinity regularization for AD detection.

In recent years, deep learning technology has made great strides on compute vision tasks, e.g. segmentation, classification, and detection. Different from the conventional methods mentioned above, deep learning-based methods can automatically find discriminative features from inputs, avoiding complex processing procedures and manually designed feature extraction operators. Inspired by the impressive performance, amounts of promising studies based on deep learning have been developed for AD prediction. As the 3D PET images can be divided into 2D slices, some scholars employed 2D CNNs to classify AD. Wang et al. [11] proposed an eight-layer convolutional neural network (CNN) with the leaky rectiﬁed linear unit and max-pooling layer for AD classiﬁcation, in which 2D slice of 3D MRI is employed as the input of CNN. Ding et al. [12] introduced the inception v3 that stacks 11 inception modules [13] into the method for AD classiﬁcation with the 4 × 4 grid images generated from the 3D PET as inputs. Liu et al. [14] proposed a classification framework based on 2D CNN and recurrent neural network (RNN) for AD classiﬁcation, in which the 2D CNN is used to capture the intraslice features, and RNN is employed to learn and integrate the interslice features. Afterwards, the ﬁnal results were obtained by fusing the prediction scores from three directions of 3D PET.

Although the mentioned methods with 2D CNNs show effectiveness in AD classification, one of the shortcomings of the methods is that the spatial information of the 3D image is not fully utilized. In order to solve this problem, CNNs with 3D kernels are developed to better utilize the spatial information. Huang et al. [15] constructed a 3D VGG variant model based on single modality for AD diagnosis and achieved multimodality detection by concatenating the multimodality features obtained from MRI and PET images. In addition, the experimental results in [15] showed that hippocampus segmentation is not necessary for improving the performance of the CNN-based classification method. Liu et al. [16] developed a CNN-based model for AD automatic diagnosis with various techniques for designing the CNN model. Zhou et al. [17] utilized a sparse-response deep belief network (SR-DBN) with extreme learning machine (ELM) to classify NC, MCI, and AD. Liu et al. [18] designed a diagnostic framework to extract complementary information from multiple inputs by using zero-masking strategy for prediction. Yee et al. [19] designed a 3D CNN-based network with residual connections for AD diagnosis, and class activation maps implicate many known regions affected by AD. Pan et al. [20] developed a multiview separable pyramid network-based classification model for AD prediction, in which the features are extracted from axial, coronal, and sagittal views of PET scans with the 3D CNN framework.

As inferred from literature, most of the existing studies for AD diagnosis aim at recognizing AD vs. NC or MCI vs. NC, which regard AD diagnosis as a binary classification problem. Due to the importance of MCI in early diagnosis of AD, the MCI should be accurately recognized from AD and NC. Thus, the three-category classification including NC, MCI, and AD is more reasonable for AD prediction. However, MCI is a transition state from NC to AD, and it is more difficult to be correctly identified compared with the identification of AD and NC. To tackle the 3-category classification, one direct way is to build a 3-category classifier for classification, but this is usually not able to achieve excellent enough performance as usual, especially for the prediction of MCI. Therefore, more attention needs to be paid on the identification of MCI than the other two categories.

Besides, there is still a big space for improving the performance in AD diagnosis of deep learning-based methods due to the limitation of scarce training samples. Since the success of deep learning is partially attributed to the training data, it is believed that a discriminative and robust deep learning-based model can be learned with a large-scale and variable dataset. However, because of the difficulties of PET image acquisition and the high cost of manual annotation, it is infeasible to obtain sufficient training data, which decreases the generalization ability in working data.

In view of the optimal property of SVM in solving binary classifications and the powerful feature extraction ability of deep CNNs, in this paper, we proposed a hybrid model integrated with CNN and SVM networks for AD prediction. The CNN model composed of 3D convolution kernels is developed to extract deep features, while the SVM [21] is utilized for classification. Moreover, an end-to-end training algorithm is developed for further fine-tuning the hybrid system. Since the SVM-based classifier is designed for binary classification, to tackle the 3-category classification problem with the proposed hybrid model, a decision fusion algorithm is proposed to fuse the results of three hybrid models for performing NC, MCI, and AD prediction, in which one network is employed for two of three-category prediction. Extensive experiments have been conducted in the work, and the experimental results show that the proposed approach achieves outstanding performance, compared with the state-of-the-art methods.

The sequel of this paper is organized as follows: Section 2 presents the detailed description of the proposed method, and Section 3 gives the experimental results and performance analysis on the database used in the work. Finally, Section 4 draws conclusions of the contributions made in the paper.

## 2. Proposed Method

### 2.1. Overall Scheme of the Proposed Method

In this paper, we proposed a hybrid model integrated with CNN and SVM networks to predict NC, MCI, and AD. The structure of the proposed model is shown in Figure 1 that consists of two modules, a feature extraction module based on CNN with 3D kernels (3DCNN), and a SVM-based classification module. Briefly, the feature extraction module is to extract deep features of the input 3D PET images and the classification module is to classify the features to get final decisions. Inspired by [16], the 3DCNN model is redesigned here in according to the purpose of this paper so as to utilize the spatial information provided by the PET images. In addition, to further improve the performance of the model with small batch sizes caused by large 3D data, instance normalization (IN) [22] is employed for normalization. Besides, channel attention [23] is also introduced into the 3DCNN to select more important features. Under the assumption of scarce annotated training data, the SVM-based classification module with the kernel function is employed to find the global structural optimal hyperplane of the training features from all the training samples.

In the training stage, the training data are first sent to the feature extraction module for classification. Then, the outputs of the global average pooling layer (GAP) of the feature extraction module shown in Figure 2 are taken as the inputs of the SVM-based classification module. Next, the parameters of the SVM are solved by the extracted features of training data. Finally, the hybrid model is trained end-to-end by the designed strategy to further optimize the parameters of the model. In the testing stage, the inputs are first sent to the 3DCNN module to extract deep features. Then, the classification results are obtained by the SVM according to the extracted features.

For early AD diagnosis, the proposed model should tackle the problem of 3-category classification. Due to the optimal classification performance for binary classifications of SVM, we divide the three-category classification problem into three binary classification problems so as to boost the performance of 3-category classification, each binary problem being solved by one hybrid model. The overall structure of this three-category classification system is shown in Figure 3, in which it consists of three branches, each binary classification being realized with one 3DCNN + SVM hybrid network. In order to obtain the final classification decision according to the three branch classifiers, a decision fusion algorithm is proposed to fuse the outputs of three 3DCNN + SVM classifiers. The details of the proposed classification system will be given in the sequel sections.

### 2.2. 3DCNN-Based Feature Extraction Module

CNN is widely used in the field of computer vision currently [24] owing to its powerful feature extraction ability. Different from conventional methods that extract features manually, CNN can automatically learn features through an end-to-end training process. In order to utilize the advantage of CNN and the spatial information of input 3D PET images, we design a 3DCNN-based feature extraction module to extract deep features. The structure of the designed 3DCNN network is described in Table 1 and Figure 2, and it is composed of 6 convolutional layers with 3D kernels to extract features, 4 max-pooling layers for downsampling, and 4 attention layers to select the informative channels. The typical 3D CNNs, such as 3D DenseNet [25] and 3D ResNet [26], usually employ large-scale kernels to compress the input in the first convolutional layer, which may lose the detailed information. To better learn the lesion feature from the 3D PET images, the first two convolutional layers involved in the model do not perform dimension reduction. The kernel size of the two layers is 1 × 1 × 1 and 3 × 3 × 3 with a stride of 1, and the number of kernels is set to 32 and 64 to extend the features, separately. Afterwards, to reduce the computational complexity, a 2 × 2 × 2 MaxPooling3D layer is employed to reduce the size of the features by half. Then, four convolutional layers, each followed by a channel attention module and a 2 × 2 × 2 MaxPooling3D layer, are adopted to learn more generalization representations. The channel attention mechanism utilized here is based on the CBAM [23] to enable the model to pay more attention to significant features. The mechanism employs multilayer perceptron (MLP) with one hidden layer to generate attention vector *W* as attention weights for feature selection, and *W* can be computed as

(1) $$\begin{array}{c} W\left(F\right)=\sigma \left(\text{MLP}\left(\text{AvgPool}\left(F\right)\right)+\text{MLP}\left(\text{MaxPool}\left(F\right)\right)\right), \end{array}$$

where *F* denotes the input feature map and *σ*(·) is the sigmoid function. The MaxPooling3D layer followed the mechanism module is to compress the deep features. Moreover, to speed up the network training and maintain excellent performance on small batch size, the IN [22] layer after each convolutional layer is introduced into the system as in [16] to conduct feature normalization. Besides, after each convolutional layer, a Rectified Linear Unit (ReLU) is utilized as the activation function to conduct nonlinear transformation, thereby preventing the network from degrading into a linear system.

To optimize the model using the annotated data, a fully connected layer after a global average pooling (GAP) layer is utilized to perform binary classification at the end of the last convolutional. Notably, the fully connected layer here is only to optimize the network to gain initial weights, and the outputs of the feature extraction module obtained after the GAP layer are used for subsequent classification.

In addition, to improve the robustness of the model against small batch size training, we update the network with the average gradient from multiple batches. Moreover, the technologies of dropout and label smoothing are employed [27, 28] as well.

### 2.3. SVM-Based Classification Module and an End-to-End Training Algorithm for CNN + SVM Model

SVM with the nonlinear kernel function is able to transform a nonlinear separable problem into a linear separable problem and then finds the structural optimal separate hyperplane that has the maximum margin between the two classes [21]. Because of the small size of annotated training data, the global optimal solution of the training data is available in the conditional that the features extracted by the feature extraction module are ﬁxed. To this end, we employ the SVM with polynomial kernel as the classification module to find the structural optimal solution from all the training data. Nevertheless, it is known that the performance of SVM depends on the support vectors. Once the CNN is trained, the support vectors are fixed. In order to further optimize the parameters of the CNN by using the optimal hyperplane obtained by SVM in the embedding feature space, an end-to-end training algorithm is developed for the proposed hybrid model. The details of the SVM-based classification module and the end-to-end training algorithm are introduced as follows.

As introduced in [21], the purpose of SVM is to find a separation hyperplane, which maximizes the distances between the margins of two kinds of categories. For *n* sample features {(**x**_*i*_, *y*_*i*_)}_*i*=1_^*n*^, **x**_*i*_ ∈ **R**^1×*d*^, **x**_*i*_={*x*_*i*_^1^, *x*_*i*_^2^,…, *x*_*i*_^*d*^}, and *y*_*i*_ ∈ {−1,1}, the objective function of SVM is defined by

(2) $$\begin{array}{c} L\left(w,b,\alpha ,\xi \right)=\frac{1}{2}{\left\|w\right\|}^{2}+C\sum_{i=1}^{n}\xi_{i}-\sum_{i=1}^{n}\left.\left[a_{i}y_{i}\left(w^{T}x_{i}+b\right)-1\right]\right\}, \end{array}$$

where **w** ∈ *R*^*d*×1^ is the coefficient vector, *b* is the bias term, *α* ≥ 0 is Lagrange multiplier, *ξ* is the slack variables, and *C* ≥ 0 is a penalty parameter used to control the degree of penalty for misclassification. To optimize the SVM by minimizing the objective function, (2) is usually solved by the following dual problem:

(3) $$\begin{array}{c} Q\left(\alpha \right)=\sum_{i=1}^{n}\alpha_{i}-\frac{1}{2}\sum_{j=1}^{n}\sum_{i=1}^{n}\left\{\alpha_{i}\alpha_{j}y_{i}y_{j}K\left(x_{i},x_{j}\right)\right\},\\ \text{Subjected to:}0\leq \alpha_{i}\leq C,\;\sum_{i=1}^{n}a_{i}y_{i}=0, \end{array}$$

where *i* and *j* ∈ 1,…, *n* and *K*(*x*_*i*_, *x*_*j*_) is the kernel function. In the paper, the polynomial kernel function is utilized as the kernel function that is defined as

(4) $$\begin{array}{c} K\left(x,x_{i}\right)={\left[\left(x\cdot x_{i}\right)+1\right]}^{q}, \end{array}$$

where *x* is the input vector, *x*_*i*_ denotes the support vector of SVM, and *q* is the order of polynomial.

For the input *x*, the decision function is defined as

(5) $$\begin{array}{c} y=\text{sign}\left(\sum_{i}\alpha_{i}y_{i}K\left(x,x_{i}\right)+b\right)=\text{sign}\left(s\right). \end{array}$$

Obviously, after solving the parameters of *α*_*i*_ and *b*, the classification result of *x* can be obtained. In the paper, the sequential minimal optimization (SMO) algorithm [29] is utilized to calculate *α*_*i*_ and *b*.

As shown in (5), a nonderivable sign function is employed to binarize the value of the linear output of SVM to obtain finally prediction. Due to that the output of sign function is 1 or −1, the influence of the linear output value *s* of SVM is ignored. In general, higher value of the output in the classification indicates higher confidence that the input belongs to the corresponding category. In addition, the BP algorithm cannot be performed by using a nondifferentiable sign function. In order to tackle the problems, a modified SVM is proposed for classification and an end-to-end training algorithm integrated with CNN and modified SVM is proposed to further optimize the hybrid model.

For the modified SVM, the sign function is replaced with a differentiable softmax-based function. Since SVM only has one output, the linear value *s* together with its opposite value, −*s*, are utilized as the inputs of softmax function. The structure of the modified SVM is shown in Figure 4, and its output can be computed as

(6) $$\begin{array}{c} y=f\left(\sum_{i=1}^{n}w_{i}K\left(x,x_{i}\right)+b\right)=f\left(s\right), \end{array}$$

where *w*_*i*_=*α*_*i*_*y*_*i*_ can be regarded as the weights of the output of *K*(*x*_*i*_, *x*), *f* (·) is the softmax function-based differentiable function, and **y** = {*y*_0_, *y*_1_} is the output of the modified SVM, in which **y** can be obtained by

(7) $$\begin{array}{c} y_{0}=q\left(x\in d_{+}\right)=\frac{e^{s}}{e^{s}+e^{-s}}, \end{array}$$

(8) $$\begin{array}{c} y_{1}=q\left(x\in d_{-}\right)=\frac{e^{-s}}{e^{s}+e^{-s}}, \end{array}$$

where *x* is the input feature, *s* is the linear output value of SVM, *q*(*x* ∈ *d*_+_) denotes the probability of *x* belonging to the positive class, and  *q*(*x* ∈ *d*_−_) denotes the probability of *x* belonging to the negative class.

The modified SVM shown in Figure 4 can be equivalent to a neural network with one hidden layer, thus the hybrid model can be trained end-to-end. In the article, the cross-entropy loss is employed to optimize the hybrid model, in which the loss function is defined as

(9) $$\begin{array}{c} H\left(p,q\right)=-\sum_{i=1}^{n}\left(p\left(x_{i}\in d_{+}\right)\log q\left(x_{i}\in d_{+}\right)\right.\\ \left.+\left(1-p\left(x_{i}\in d_{+}\right)\right)\log\left(1-q\left(x_{i}\in d_{+}\right)\right)\right), \end{array}$$

where *p* is the label function that is defined as *p*=1 if *x* ∈ positive sample; else, *p* = 0; and *n* indicates the total number of the training samples.

Equations (7) and (8) can also be represented by

(10) $$\begin{array}{c} q\left(x\in d_{+}\right)=\frac{1}{1+e^{-2s}},\\ q\left(x\in d_{-}\right)=\frac{1}{1+e^{2s}}. \end{array}$$

Obviously, for a positive class feature, only *s* tends to positive infinity, *q*(*x* ∈ *d*_+_) equals to 1, and loss function *H* (*p*, *q*) tends to 0. Since *s* is positively related to the distance from *x* to the hyperplane of SVM, the larger *s* means the greater distance between *x* and the hyperplane. For a negative class feature, the loss function *H* (*p*, *q*) tends to 0 when *s* tends to negative infinity. Thus, the loss function can be utilized to optimize the features of CNN and further increase the margin between the two classes.

The optimization of SVM is to find the optimal hyperplane from all training samples, which is different from the backwardpropagation (BP) algorithm-based optimization of 3DCNN. In order to jointly optimize the hybrid system with the BP algorithm and maintain the optimal structure of SVM, the parameters of the SVM are not adjusted in the process of optimizing CNN with the BP algorithm. After CNN converged, the parameters of SVM are re-calculated by the SMO algorithm to find the new separate hyperplane for further optimization.

Details for these operation steps are as follows:

- Initialize a 3DCNN and a SVM to be trained, and divide the PET dataset into 3 subsets (training set, verification set, and test set)
- Train the 3DCNN by using the samples in the training set until converged, and then, use the converged 3DCNN to extract the feature vector output from its last pooling layer using all the samples in the training set and in the verification set as input
- Train the SVM by using the extracted feature vectors as training samples obtained by using the input samples in the training set in Step (ii), until the SVM converged
- Construct a 3DCNN + SVM network using the trained 3DCNN and SVM, and replace sign function with softmax function as described in (7) and (8)
- Fine-tune the 3DCNN + SVM network by using the samples both in the training set and in the verification set and the loss function computed according to (9), with the weights of the SVM ﬁxed (without updated), until the 3DCNN converged basically
- Re-train the SVM by using the extracted feature vectors output from the 3DCNN obtained in Step (v) without updating the 3DCNN, until the SVM converged basically
- Repeat the Steps (iv)–(vi), until the whole 3DCNN + SVM network converged
- Test the trained 3DCNN + SVM network by using the samples in the test set

### 2.4. Decision Fusion Algorithm of Three Binary Classifiers

At present, most of the existing studies related to AD aim to solve binary classiﬁcation problems, such as AD vs. NC and MCI vs. NC. However, in practical applications, a robust 3-category classiﬁcation model is crucial for the early diagnosis of AD as mentioned above. Generally, this problem can be well solved directly by a 3-category classifier, but it may not be suitable for AD prediction with a simple 3-category classifier as the MCI is hard to be accurately identified from AD and NC. Since the proposed SVM-based classification module can achieve global optimal structure solutions for binary classification on the training data, 3-category classification task can be solved by using three hybrid models with the proposed decision fusion algorithm.

As shown in Figure 3, three 3DCNN_i_ + SVM_*i*_ networks (*i* = 1, 2, and 3) are built up to cope with the three-category classification with one network for solving two of three-category classification. Before making a final decision, three 3DCNN + SVM hybrid networks need to be trained in advance for performing the binary classifications of AD vs. NC, MCI vs. NC, and AD vs. MCI. Afterwards, for a 3D PET image to be classified, it is first fed into the three 3DCNN_i_ + SVM_i_ networks (*i* = 1, 2, and 3) respectively, and then, outputs of the three classification models can be obtained. In order to use the results of the three classifiers effectively, in the paper, we design a decision fusion algorithm as follows to get the final decision:

(1) If the results of two classification models belong to the same category, the category is regarded as the final classification result
(2) If all the three classification results are different, the final decision is made according to the absolute value, *|s*_*i*_*|*, of the linear output of the SVM_*i*_ (*i* = 1, 2, and 3) as follows:
  (11) $$\begin{array}{c} k=\arg\underset{i}{\max}\left(\left|s_{i}\right|\right). \end{array}$$
Then, final classification result is selected as the binary classification result of the *k*th 3DCNN + SVM network (i.e., the output of the SVM_*k*_).

## 3. Experiments

### 3.1. Database and Data Preprocessing

In order to evaluate the proposed method in AD prediction, the ^18^F-Fluorodeoxyglucose positron emission tomography (^18^F-FDG PET : PET) data obtained from the Alzheimer's Disease Neuroimaging Initiative (ADNI) database [30] launched in 2003 are utilized in the paper, in which ADNI has been committed to tracking the progress of AD through biomarkers and clinical assessments. By identifying sensitive and specific markers of early AD progression in the database provided by the participants at different time, it can help researchers and clinicians develop new treatments, monitor the effectiveness, and reduce the cost of clinical trials.

In this work, we adopt 2706 3D PET images from 959 ADNI participants, including 267 AD subjects, 340 MCI subjects, and 352 NC subjects.  Table 2 presents the demographic details of the studied subjects in the work, where MMSE is the abbreviation of the Mini-Mental State Examination. The PET images are first preprocessed by performing image registration, spatial normalization, intensity normalization, and image smoothing. Then, the voxels outside the brain are removed from the PET images, and the images are cropped to a size of 80 × 100 × 76.

### 3.2. Implementation Settings and Evaluation Indexes

All the models and algorithms adopted in the work have been implemented, and all the experiments are conducted by using Python on a CPU + GPU platform with the CPU of Intel ®Core™ i77700@3.60 GHz and the GPU of NVIDIA GeForce GTX 1080Ti.

In the experiment, five-fold cross-validation is performed, where the dataset is divided into 5 equal parts in which 1 part is used as the testing data and 4 parts are used as training data with 1 part of them as verification data. And, the experiments are conducted 5 times in turn, and the mean values of the results of 5 trials are used as final indexes of the method. The data are strictly divided according to patient's IDs to ensure that the image samples of the same person will not be put into different datasets, i.e., the PET images of one participant are put into only one part in the data partition to avoid data leakage. The stochastic gradient descent (SGD) algorithm is utilized to minimize the loss function in training the proposed model. The batch size is set to 4, and the weights of the network are updated every four batches for better convergence in the training process.

To better evaluate the performance of the proposed method and state-of-the-art methods, 4 technical indexes [20] are employed for evaluation, including accuracy (ACC), sensitivity (SEN), speciﬁcity (SPE), and AUC (area under ROC curve). The ACC, SEN, and SPE are the proportion of correct predictions among all samples, positive samples, and negative samples, respectively. Each of the indexes is identified as

(12) $$\begin{array}{c} \text{ACC}=\frac{\text{TP}+\text{TN}}{\text{TP}+\text{TN}+\text{FP}+\text{FN}},\\ \text{SEN}=\frac{\text{TP}}{\text{TP}+\text{FN}},\\ \text{SPE}=\frac{\text{TN}}{\text{TN}+\text{FP}}, \end{array}$$

where TP, FP, TN, and FN separately indicate the true positive, false positive, true negative, and false negative. The AUC is obtained by computing the area under the receiver operating characteristic curve (ROC) which is the curve to describe the relationship between the true positive rate (TPR) and the false positive rate (FPR) under varied threshold settings. Obviously, the higher result stands for better performance.

### 3.3. Evaluation of the Proposed Method Applied to Binary Classification

In this section, experiments are conducted for the proposed 3DCNN + SVM classification method and also for the other state-of-the-art methods, respectively. The methods proposed in the cited literature were originally designed for solving binary classification problems, such as the prediction of AD vs. NC or MCI vs. NC. For our proposed method, since a single 3DCNN + SVM model with end-to-end training is also proposed for solving a binary classification problem, we just need to use a single 3DCNN + SVM network to perform the classification without needing three such networks.

Aiming to better evaluate the generalization performance of the proposed method and the state-of-the-art ones, we test the approaches on both training and testing sets. Tables 3–5 present the experimental results implemented on the data of AD vs. NC, MCI vs. NC, and AD vs. MCI, respectively. Since the experimental results given in the cited literature were obtained by using different data partitions under different experiment settings, in order to make a fair comparison, the methods without “^*∗*^” are implemented by using the same PET data under the same experiment settings as in ours in the paper; meanwhile, the results of the methods with “^*∗*^” are cited by the corresponding reference. From the results shown in the tables, one can see that the proposed method generally performs better than the other ones, and its effectiveness can be confirmed by the experiments.

In addition, Figure 5 displays the comparisons of the ROC curves on AD vs. NC, MCI vs. NC, and AD vs MCI. From the figure, we can observe that the proposed method achieves the best AUC compared with the mentioned state-of-the-art methods and proves the robustness and effectiveness of the hybrid model.

### 3.4. Evaluation of the Proposed Method Applied to 3-Category Classification

As mentioned before, in order to solve the early prediction of AD symptoms, a hybrid 3-category classification system is developed by integrating three binary 3DCNN + SVM classifiers with an optimal decision fusion scheme. In this section, we present the experimental results to evaluate this 3-category classification system by using the 3D PET images from MCI, AD, and NC subjects. In order to demonstrate the effectiveness of the proposed method, the “CNN + BGRU” method introduced in [14] and the “ADCNN” model proposed by Liu et al. [16] are implemented in the paper for comparison. In this work, we re-implement the CNN-based state-of-the-art methods and train and test by using the same 3D PET images as used in the paper.  Table 6 shows the experiment results on training and testing sets, in which the experimental results of “3DCNN” are also included that are obtained by using a three-dimensional CNN network with the same structure as the 3DCNN shown in Figure 2 but adjusting the number of the output fully connected layer nodes from 2 to 3. This “3D-CNN” model is also trained and tested by using the same data as the other models and also used for performance comparison in the experiment.

From the results shown in Table 6, it can be seen that the proposed hybrid 3-category classification system obtains a signiﬁcant improvement on all the four evaluation indexes, compared with the others. According to the results of Tables 3–6, it implies that the proposed method not only achieves excellent performance in binary classification tasks but also outperforms the other methods in three category classification by applying the proposed decision strategy with three proposed binary classifiers.

### 3.5. Ablation Experiments of the CNN + SVM Hybrid Model with End-to-End Training Algorithm

For the proposed method, the SVM is employed to replace the fully connected layer of the proposed 3DCNN as the classifier, and an end-to-end algorithm is developed to optimize the hybrid model.

In order to compare the performance of the improvement and, meanwhile, validate the effectiveness of the integration, we conduct ablation experiments to evaluate the proposed improvement including the SVM-based classifier and the end-to-end algorithm. Tables 7–9 show the ablation results of the proposed module evaluated on the data of AD vs. NC, MCI vs. NC, and AD vs. MCI on both training and testing sets, respectively. In order to make a fair comparison, the 3DCNN network illustrated in Figure 2 is employed as the baseline for further comparison. To assess the effects of the SVM-based classifier, in this section, the results of “3DCNN + SVM” are obtained by directly combining the baseline with an SVM without the proposed end-to-end algorithm, i.e., the two modules are trained separately. From the results of the three binary-category classification tasks, the “3DCNN + SVM” can give relatively better overall performance than the baseline, which proves the effectiveness of the SVM-based classifier on AD prediction with scarce training data. To further optimize the hybrid model, the end-to-end algorithm is developed to fine-tune the 3DCNN model. The results of “3DCNN + SVM + E2E” are obtained by using the proposed end-to-end training methods. With the assistance of the end-to-end algorithm, the performance of the proposed module is improved again on the indexes of ACC, SEN, SPE, and AUC.  Figure 6 displays the comparisons of the ROC curves on AD vs. NC, MCI vs. NC, and AD vs. MCI for the above ablation experiments, which further proves the effectiveness of the proposed implementations for AD prediction. Therefore, according to the ablation studies, the proposed SVM-based classifier and the end-to-end algorithm play an important role in boosting the performance of the baseline on AD diagnosis.

In addition, we also visualize the features extracted by the outputs after the global average pooling layer of 3DCNN before and after end-to-end training, and the visualization results are shown in Figures 7–9 . From the results, it can be seen that the features in visual are easier to be recognized after end-to-end training, which confirms the feasibility of the proposed end-to-end algorithm.

### 3.6. Ablation Studies of the Implemented 3DCNN

In this section, we validate the effectiveness of the key technologies employed in the 3DCNN model, mainly including the channel attention mechanism and the instance normalization method.  Table 10 shows the ablation results on AD vs. NC prediction. The “3DCNN w/o Atten” is the model that removes the channel attention mechanism from the designed 3DCNN, and the “3DCNN with Atten” is the proposed 3DCNN model shown in Figure 2. As can be seen, the model with channel attention is superior to the model without the attention mechanism in the four indexes, which shows that the measure is effective for improving the recognition accuracy.

In addition, due to the small batch size caused by a large scale of image data, the instance normalization (IN) is employed to replace the typical batch normalization (BN) for the designed 3DCNN model. The comparison experiments are conducted in Table 11, in which the 3DCNN with BN is the model that uses BN as the normalization function, and the 3DCNN with IN is the proposed 3DCNN model. It can be seen from the results that the performance of the 3DCNN is improved after replacing BN with IN, and the sensitivity is the most obvious. As a result, from the results in Tables 10 and 11, the measures introduced into the proposed 3DCNN model are helpful in improving the performance of the model.

## 4. Summary and Further Working Direction

In this paper, we proposed a new classiﬁcation system for early automatic diagnosis of AD symptoms based on 3DCNN and SVM, in which the original 3-category classification problem is divided into three binary classification problems; each binary classification is realized with a 3DCNN + SVM model. Furthermore, an end-to-end learning algorithm is developed for training the 3DCNN + SVM networks, and an optimal decision fusion scheme is proposed to fuse the outputs of three 3DCNN + SVM classifiers based on the criteria of majority voting. By using these methods, the advantages of both CNN and SVM models can be fully utilized; thus, the overall performance of the system can be significantly improved. Experimental results obtained in the paper confirm the effectiveness of the proposed approach that outperforms the existing start-of-the-art methods in terms of the class accuracy, sensitivity, specificity, and area under ROC.

It is noticed that, from the experimental results obtained in the paper, the classification performance of MCI samples still leaves some room for further improvement, and the correct identification of this category samples is crucial for the early diagnosis of AD. Therefore, a more effective method is needed to be developed to overcome this shortage, which will be the future research direction of the paper.

## Figures and Tables

**Figure 1:** Block diagram of the scheme for the 3DCNN + SVM method.

**Figure 2:** The structure of the proposed feature extraction module.

**Figure 3:** Block diagram of the overall scheme for three-category classification.

**Figure 4:** The equivalent neural network of SVM with the nonlinear kernel function.

**Figure 5:** ROC curves of the proposed method and state-of-the-art methods on AD vs. NC, MCI vs. NC, and AD vs. MCI. (a) AD vs. NC. (b) MCI vs. NC. (c) AD vs. MCI.

**Figure 6:** ROC curves of the ablation experiments on 3DCNN + SVM. (a) AD vs. NC. (b) MCI vs. NC. (c) AD vs. MCI.

**Figure 7:** The visualization results of the features extracted from the 3DCNN before and after the end-to-end training algorithm on AD vs. NC. (a) The results before end-to-end training. (b) The results after end-to-end training.

**Figure 8:** The visualization results of the features extracted from the 3DCNN before and after the end-to-end training algorithm on MCI vs. NC. (a) The results before end-to-end training. (b) The results after end-to-end training.

**Figure 9:** The visualization results of the features extracted from the 3DCNN before and after the end-to-end training algorithm on AD vs. MCI. (a) The results before end-to-end training. (b) The results after end-to-end training.

**Table 1:** The architecture of 3DCNN designed in the paper.

Layer ID	Layer	Kernel number	Kernel size/stride	Output size
0	Input			1 × 80 × 100 × 76
1	Conv1	32	(1, 1, 1)/1	32 × 80 × 100 × 76
2	Conv2	64	(3, 3, 3)/1	64 × 80 × 100 × 76
3	MaxPool3D		(2, 2, 2)/2	64 × 40 × 50 × 38
4	Conv3	128	(3, 3, 3)/1	128 × 40 × 50 × 38
5	Attention			128 × 40 × 50 × 38
6	Maxpool3D		(2, 2, 2)/2	128 × 20 × 25 × 19
7	Conv4	256	(3, 3, 3)/1	256 × 20 × 25 × 19
8	Attention			256 × 20 × 25 × 19
9	Maxpool3D		(2, 2, 2)/2	256 × 10 × 12 × 9
10	Conv5	512	(3, 3, 3)/1	512 × 10 × 12 × 9
11	Attention			512 × 10 × 12 × 9
12	Maxpool3D		(2, 2, 2)/2	512 × 5 × 6 × 4
13	Conv6	512	(3 × 3 × 3)/1	512 × 3 × 4 × 2
14	GAP			512 × 1 × 1 × 1
15	Flatten			512
16	FC			2

**Table 2:** Demographic characteristics of the studied subjects.

Diagnosis	Number	Age	Gender (F/M)	MMSE
AD	514	75.98 ± 7.62	305/209	19.26 ± 5.64
MCI	1247	76.47 ± 7.54	809/438	22.83 ± 6.56
NC	945	76.99 ± 5.95	544/405	27.83 ± 3.63

**Table 3:** Evaluation of the proposed 3DCNN + SVM with E2E applied to binary classification of AD vs. NC samples (%).

Method	Training set				Testing set			
	ACC	SEN	SPE	AUC	ACC	SEN	SPE	AUC
Gray [6]^*∗*^	—	—	—	—	81.60	82.7	80.4	90.0
Lu [10]^*∗*^	—	—	—	—	89.44	88.89	90.0	—
Silveira [8]^*∗*^	—	—	—	—	**90.97**	—	—	—

Ding et al. [12]	98.92	99.49	98.61	98.95	86.27	86.97	85.78	90.50
Liu et al. [14]	98.61	**99.59**	98.07	99.84	89.31	87.50	90.32	92.96
Huang et al. [15]	**99.21**	99.43	98.48	99.35	88.68	87.74	89.17	91.98
Proposed	99.19	99.39	**99.54**	**99.88**	**90.82**	**91.29**	**90.59**	**93.75**

**Table 4:** Evaluation of the proposed 3DCNN + SVM with E2E applied to binary classification of MCI vs. NC samples (%).

Method	Training set				Testing set			
	ACC	SEN	SPE	AUC	ACC	SEN	SPE	AUC
Gray [6]^*∗*^	—	—	—	—	70.20	73.80	62.30	73.0
Lu [10]^*∗*^	—	—	—	—	**79.63**	—	—	—
Silveira [8]^*∗*^	—	—	—	—	70.00	46.96	**80.44**	—

Ding et al. [12]	98.70	98.05	99.55	99.43	72.37	74.70	69.31	79.19
Liu et al. [14]	99.04	98.52	99.74	99.73	73.80	73.16	74.69	80.45
Huang et al. [15]	98.30	97.72	99.09	**99.97**	73.52	75.50	70.90	79.65
Proposed	**99.54**	**99.26**	**99.90**	99.88	**76.68**	**77.80**	**75.57**	**82.39**

**Table 5:** Evaluation of the proposed 3DCNN + SVM with E2E applied to binary classification of AD vs. MCI samples (%).

Method	Training set				Testing set			
	ACC	SEN	SPE	AUC	ACC	SEN	SPE	AUC
Gray [6]^*∗*^	—	—	—	—	68.2	58.3	73.0	70.0
Lu [10]^*∗*^	—	—	—	—	—	—	—	—
Silveira [8]^*∗*^	—	—	—	—	70.0	—	—	—

Ding et al. [12]	92.39	97.50	90.29	98.59	71.19	68.52	72.36	77.28
Liu et al. [14]	96.10	**99.93**	94.52	99.18	73.79	**75.00**	73.28	79.16
Huang et al. [15]	96.09	99.66	94.53	99.39	73.83	74.93	73.42	78.53
Proposed	**98.45**	99.24	**97.31**	**99.91**	**74.29**	70.78	**75.48**	**80.11**

**Table 6:** Evaluation of the proposed method applied to 3-category classification in terms of ACC (%).

Method	Training set				Testing set			
	AD	MCI	NC	Average	AD	MCI	NC	Average
Cabral et al. [9]^*∗*^	—	—	—	—	—	—	—-	66.78
3DCNN	**99.85**	98.62	99.89	**99.45**	65.63	62.12	70.43	65.66
CNN + BGRU [14]	97.75	**99.89**	99.86	99.17	58.65	66.22	68.28	65.53
ADCNN [16]	99.81	98.35	**99.99**	99.38	65.16	63.25	68.63	65.44
Proposed	99.17	97.83	99.37	98.79	**73.42**	**67.86**	**72.28**	**71.19**

**Table 7:** Ablations studies of the proposed 3DCNN + SVM model applied to binary classification of AD vs. NC (%).

Method	Training set				Testing set			
	ACC	SEN	SPE	AUC	ACC	SEN	SPE	AUC
3DCNN	**99.50**	**99.72**	99.39	**99.97**	89.83	90.94	89.26	92.68
3DCNN + SVM	98.62	99.01	98.40	99.95	90.20	90.34	90.19	93.36
3DCNN + SVM + E2E	99.19	99.39	**99.54**	99.88	**90.82**	**91.29**	**90.59**	**93.75**

**Table 8:** Ablations studies of the proposed 3DCNN + SVM model applied to binary classification of MCI vs. NC (%).

Method	Training set				Testing set			
	ACC	SEN	SPE	AUC	ACC	SEN	SPE	AUC
3DCNN	**99.80**	**99.66**	99.55	**99.99**	75.04	75.54	72.97	79.74
3DCNN + SVM	98.35	98.30	98.41	**99.99**	75.58	76.42	74.41	80.80
3DCNN + SVM + E2E	99.54	99.26	**99.90**	99.88	**76.68**	**77.80**	**75.57**	**82.39**

**Table 9:** Ablations studies of the proposed 3DCNN + SVM model applied to binary classification of AD vs. MCI (%).

Method	Training set				Testing set			
	ACC	SEN	SPE	AUC	ACC	SEN	SPE	AUC
3DCNN	98.37	**99.73**	**97.72**	99.81	73.56	**73.84**	73.51	77.82
3DCNN + SVM	97.72	99.43	96.80	99.84	73.95	71.88	74.89	78.75
3DCNN + SVM + E2E	**98.45**	99.24	97.31	**99.91**	**74.29**	70.78	**75.48**	**80.11**

**Table 10:** Ablations studies of the channel attention mechanism on AD vs. NC (%).

Method	Training set				Testing set			
	ACC	SEN	SPE	AUC	ACC	SEN	SPE	AUC
3DCNN w/o Atten	98.74	**99.88**	99.12	99.78	89.41	90.55	88.83	91.92
3DCNN with Atten	**99.50**	99.72	**99.39**	**99.97**	**89.83**	**90.94**	**89.26**	**92.68**

**Table 11:** Comparison of different normalization functions of SVM on AD vs. NC (%).

Method	Training set				Testing set			
	ACC	SEN	SPE	AUC	ACC	SEN	SPE	AUC
3DCNN with BN	99.04	99.21	**99.48**	99.92	89.36	89.68	89.16	91.96
3DCNN with IN	**99.50**	**99.72**	99.39	**99.97**	**89.83**	**90.94**	**89.26**	**92.68**

## Data Availability

The publicly available ADNI dataset [30] can be downloaded through the website at http://adni.loni.usc.edu/.
